# Leukemia Inhibitory Factor Facilitates Self-Renewal and Differentiation and Attenuates Oxidative Stress of BMSCs by Activating PI3K/AKT Signaling

This article has been retracted.

**DOI:** 10.1155/2022/5772509

**Published:** 2022-09-05

**Authors:** Youde Liang, Ruiping Zhou, Xin Liu, Lin You, Chang Chen, Xiaoling Ye, Wei Wei, Jie Liu, Jiawei Dai, Kaixiong Li, Xiangxiang Zhao

**Affiliations:** ^1^Department of Stomatology, Southern University of Science and Technology Yantian Hospital, Shenzhen, Guangdong, China; ^2^Department of Neurology, Changhai Hospital, Naval Medical University, Shanghai, China

## Abstract

**Objective:**

Transplantation of bone marrow-derived mesenchymal stem cells (BMSCs) remains a hopeful therapeutic approach for bone defect reconstruction. Herein, we investigated the effects and mechanisms of leukemia inhibitory factor (LIF) in the function and viability of hypoxic BMSCs as well as bone defect repair.

**Methods:**

The effects of LIF on apoptosis (flow cytometry, TUNEL staining), mitochondrial activity (JC-1 staining), proliferation (colony formation, EdU staining), and differentiation (CD105, CD90, and CD29 via flow sorting) were examined in hypoxic BMSCs. LIF, LIFR, gp130, Keap1, Nrf2, antioxidant enzymes (SOD1, catalase, GPx-3), bone-specific matrix proteins (ALP, BSP, OCN), PI3K, and Akt were detected via immunoblotting or immunofluorescent staining. BMSCs combined with biphasic calcium phosphate scaffolds were implanted into calvarial bone defect mice, and the therapeutic effect of LIF on bone defect was investigated.

**Results:**

Hypoxic BMSCs had increased apoptosis and oxidative stress and reduced mitochondrial activity. Additionally, LIF, LIFR, and gp130 were upregulated and PI3K/Akt activity was depressed in hypoxic BMSCs. Upregulated LIF alleviated apoptosis and oxidative stress and heightened mitochondrial activity and PI3K/Akt signaling in hypoxic BMSCs. Additionally, LIF overexpression promoted self-renewal and osteogenic differentiation of BMSCs with hypoxic condition. Mechanically, LIF facilitated self-renewal and differentiation as well as attenuated oxidative stress of BMSCs through enhancing PI3K/AKT signaling activity. Implantation of LIF-overexpressed BMSC-loaded BCP scaffolds promoted osteogenesis as well as alleviated oxidative stress and apoptosis through PI3K/Akt signaling.

**Conclusion:**

Our findings demonstrate that LIF facilitates self-renewal and differentiation and attenuates oxidative stress of BMSCs by PI3K/AKT signaling.

## 1. Introduction

Bone defects caused by various traumas and diseases have become one of the most common clinical diseases [1]. At present, bone transplantation is the main method to solve the repair of bone defects [2]. Small-scale bone defects can achieve favorable clinical efficacy, but the treatment of large-scale bone defects, especially those complicated by infection, tumor, systemic metabolic, and vascular diseases, is still a clinical issue [3]. Therefore, to reduce surgical complexity and accelerate bone healing, innovative therapies are urgently needed. Tissue engineering techniques consisting of seed cells, scaffold materials, and growth factors play a key role in inducing regenerative repair of damaged tissues and organs [4]. Among the three basic elements of tissue engineering techniques, seed cells are essential for initiating tissue regeneration [5]. With the deepening of tissue engineering research, the importance of mesenchymal stem cells in tissue regeneration has received more and more attention [6]. However, stem cells or transplanted cells chemotactically derived from blood or bone marrow undergo apoptosis due to the release of a large number of inflammatory mediators and proapoptotic factors (local hypoxia, acidosis, accumulation of metabolites, tissue necrosis, oxidative stress, etc.) [7]. Bone marrow-derived mesenchymal stem cells (BMSCs) are one of the important cells involved in bone formation and angiogenesis. Studies have shown that human mesenchymal stem cells implanted in healthy adult nude mice can survive and maintain their own activity for at least 6 weeks [8]. However, Zhang et al. found that BMSCs die on a large scale after 3 days in hypoxic environment [9]. Yuan et al. also observed a sharp decrease in the number of BMSCs within 1 month after composite implantation with a stent [10]. BMSCs begin to die within 3 days of implantation into the ectopic osteogenic site and are barely detectable at 14 days [11]. Our previous study also found that BMSCs undergo significant apoptosis under hypoxic environment [12]. Therapeutic applications of BMSCs are limited due to the sensitivity to oxidative stress, leading to apoptosis of transplanted BMSCs in damaged bone areas [13]. Activation of PI3K/Akt signaling protects the survival and differentiation of BMSCs from oxidative stress [13]. RNA modification is a posttranscriptional mechanism, which controls gene expression and RNA metabolism [14]. The crosstalk between RNA modification and oxidative stress has been investigated in various human diseases [15]. Additionally, RNA modification exerts a crucial role in differentiation of BMSCs [16]. Enhancing BMSC function is a critical step in optimizing stem cell-mediated bone repair. The enhanced proliferative capacity enables BMSCs to expand in vitro to sufficient numbers for clinical transplantation. Additionally, after transplantation, BMSCs continue to proliferate and migrate to the injury site and differentiate into osteoblasts or secrete trophic factors to stimulate target cells. Hence, to modify BMSCs in enhancing their functions remains the main focus of recent studies on stem cell-mediated bone defect repair.

Leukemia inhibitory factor (LIF) belongs to the IL-6 family and is a natural multifunctional cytokine in the body [17]. Many tissues and cells in the human body can secrete LIF spontaneously or be induced to do so [18]. Studies have shown that LIF is an important factor in maintaining the survival and self-renewal of stem cells [19]. In vivo experiments found that LIF in a hypoxic microenvironment promotes bone development and bone repair [20]. In the study of myocardial infarction by Berry et al., they found that in the process of fighting myocardial ischemia, LIF maintains the survival and antiapoptosis of myocardial cells by activating downstream signaling pathways, related to the protection of bone marrow stem cell chemotaxis to the infarcted area [20]. The exogenous injection of LIF at the site of myocardial infarction reduces the apoptosis index of myocardial cells and protects the structure and function of cardiac tissue. LIF inhibits myocardial cell apoptosis by activating the myocardial LIF/LIFR/STAT3 signaling pathway in myocardial infarction rats [21]. In bone repair studies, after knocking out the LIF gene, fetal bone mass is reduced by 40% [22]. Our previous study found that hypoxia can induce upregulation of LIF expression in alveolar bone formation in a rat periodontal augmentation animal model (a classic model of persistent hypoxia) [23]. In addition, limited evidence demonstrates that LIF protects photoreceptor cone cells from oxidative stress injury via activation of the JAK/STAT3 pathway [24].

In this study, we found that in the bone defect environment, hypoxia activated LIF and thus activated the downstream signaling pathway PI3K/AKT, ameliorated the inhibitory effect of hypoxia-induced internal environment disturbance on bone growth, maintained BMSC survival and self-renewal and inhibited oxidative stress, and promoted osteogenic differentiation.

## 2. Materials and Methods

### 2.1. Isolation and Culture of BMSCs

C57BL/6 male mice aged 4-5 weeks weighing 16 ± 2 g (Laboratory Animal Center of Sun Yat-sen University, China) were utilized for isolating BMSCs. After the mice were sacrificed, the bilateral femurs of the rats were taken out under sterile conditions. The obtained femur was placed in PBS solution containing penicillin-streptomycin to remove residual blood and soft tissue fragments. The muscles and aponeurosis attached to the bone surface were carefully removed with a sterile scalpel and ophthalmic forceps. Ophthalmic scissors were used to remove the sacrum at both ends to expose the medullary cavity. The cells in the bone marrow cavity were washed out with *α*-MEM (Sigma-Aldrich, USA). The cell suspension was collected in a 15 mL centrifuge tube, centrifuged at 1000 rpm for 5 min at room temperature, and the supernatant was discarded after centrifugation. 7 mL freshly prepared *α*-MEM with 10% FBS was used for resuspending a single cell suspension that was inoculated into a 75 cm^2^ cell culture flask. BMSCs were placed in a 5% CO_2_, 95% air, and 100% humidity incubator at 37°C. After 72 h, the medium was changed to remove nonadherent cells every 2 days. BMSCs were passaged when they reached 80%-90% confluence. The third-generation BMSCs were used for subsequent experiments.

### 2.2. Flow Sorting

BMSCs were digested with 0.25% trypsin to collect 4 × 10^5^ cells, centrifuged at 1000 rpm for 4 min at room temperature. After discarding the supernatant, single cell suspension was prepared. Afterwards, BMSCs were incubated with monoclonal antibodies of cell surface antigens containing CD29-PE (ab218273, Abcam, USA), CD44-PE (ab23396), CD90-APC (ab25322), CD105-PE/Cy7 (ab272352), CD146-FITC (ab78451), and CD45-FITC (ab27287) on the ice in the dark for 30 min. After centrifuging at 1000 rpm for 5 min, the supernatant was discarded. Afterwards, the cells were resuspended in 500 *μ*L PBS and examined utilizing a FACSCalibur flow cytometer (BD Biosciences, USA).

### 2.3. Hypoxic Treatment and Transfection

For hypoxic treatment, BMSCs were cultured in an environment of 5% CO_2_, 1% O_2_, and 94% N_2_ for 10 days, with normoxia as controls. BMSCs that stably overexpressed LIF were conducted through transducing retroviral LIF expression vectors (Promega, USA). To construct BMSCs that stably depleted LIF, lentiviral siRNA vectors (Promega) targeting LIF were transduced into BMSCs. The infected BMSCs were chosen utilizing 2 mg/L puromycin for 14 days. PI3K/Akt signaling was activated by 30 *μ*M agonist 740Y-P (R&D Systems, UK) and blocked by 50 *μ*M inhibitor LY294002 (R&D Systems).

### 2.4. Flow Cytometry

BMSCs were washed with PBS as well as resuspended in 500 *μ*L of 1x Annexin-binding buffer (Beyotime). Afterwards, incubation with Annexin V-FITC and PI staining was implemented at room temperature in the dark for 10 min. The samples were immediately analyzed using flow cytometry. Apoptotic cells were examined with a FACSCalibur flow cytometer (BD Biosciences, USA).

### 2.5. TUNEL Staining

BMSCs were immersed utilizing 50 *μ*L TUNEL reaction reagent (Solarbio, China) at 37°C for 1 h. Afterwards, incubation with DAPI was conducted at 37°C for 30 min. Being washed with PBS, TUNEL-positive cells were captured under a fluorescence microscope (Olympus).

### 2.6. JC-1 Staining

Mitochondrial membrane potential was examined with a JC-1 kit (Merck, Germany). BMSCs were exposed to 2 *μ*M of JC-1 for 30 min in the dark at 37°C. Being washed with PBS, images were captured utilizing a fluorescence microscope (Olympus).

### 2.7. Immunoblotting

Protein separation was implemented through 12% SDS-PAGE, along with transference to PVDF membrane (Millipore, USA) as well as incubation with defatted milk. Afterwards, the PVDF membrane was subjected to immunoblotting following the indicated primary antibodies: Kelch-like ECH-associated protein 1 (Keap1; 1 : 500; ab119403; Abcam), nuclear factor-erythroid 2-related factor 2 (Nrf2; 1 : 200; ab62352), LIF (1 : 1000; ab113262), LIFR (1 : 1000; ab232877), gp130 (1 : 1000; ab259927), PI3K (1 : 1000; ab32089), p-PI3K (1 : 500; ab182651), AKT (1 : 500; ab8805), p-AKT (1 : 500; ab38449), hypoxia-inducible factor 1*α* (HIF-1*α*; 1 : 100; ab51608), superoxide dismutase 1 (SOD1; 1 : 5000; ab51254), catalase (1 : 1000; ab52477), glutathione peroxidase 3 (GPx-3; 1 : 1000; ab256470), and GAPDH (1 : 2000; ab59164). Incubation with a secondary antibody was implemented for 1 h. Protein was developed with an enhanced chemiluminescence approach.

### 2.8. Immunofluorescent Staining

BMSCs were washed with precooled PBS, followed by fixation with 4% paraformaldehyde for 10 min as well as permeability with 0.25% Triton-X100 for 15 min at room temperature. Afterwards, blockage with 1% bovine serum albumin was implemented for 60 min, along with incubation with primary antibody of LIF (1 : 100; ab113262, Abcam), LIFR (1 : 100; ab232877), alkaline phosphatase (ALP; 1 : 200; ab224335), bone sialoprotein (BSP; 1 : 200; ab270605), and osteocalcin (OCN; 1 : 200; ab198228) at 4°C overnight as well as Alexa Fluor® 488- (1 : 200; ab150077; Abcam) or Alexa Fluor® 594- (1 : 200; ab150080; Abcam) conjugated secondary antibody for 1 h. Thereafter, BMSCs were stained with DAPI for 15 min. Images were captured utilizing a fluorescence microscope (Olympus, Japan).

### 2.9. Colony Formation Assay

BMSCs were seeded onto 6-well culture plates (5 × 10^5^ cells/well). *α*-MEM was changed every 2 days. Colonies were fostered for 14 days in *α*-MEM. Being fixed by 4% paraformaldehyde, the medium was discarded and BMSCs were stained utilizing 0.1% crystal violet.

### 2.10. EdU Staining

Incubation of BMSCs with 50 *μ*M EdU-labeling medium was implemented for 2 h, along with fixation utilizing 4% paraformaldehyde for 30 min. Thereafter, BMSCs were exposed to 2 mg/mL glycine for 5 min, followed by staining with 100 *μ*L Apollo® staining reagent for 30 min. After permeabilizing by 0.5% Triton X-100 for 10 min, incubation with DAPI staining was conducted. EdU-labeled BMSCs were captured utilizing a fluorescence microscope (Olympus, Japan).

### 2.11. Establishment of Calvarial Bone Defect Murine Models

Eight-week-old C57BL/6 male mice weighing 20-25 g (Laboratory Animal Center of Sun Yat-sen University) were randomized to eight groups (10 each group). After making a 1.0 cm sagittal incision, the calvarium was exposed, and two defects were made on the skull through drilling a 4 mm hole with a trephine burr. The control mice did not receive any treatment. Bone defect mice were implanted by BCP scaffolds with LIF-overexpressed, 740Y-P, or LY294002 BMSCs. The incisions were closed with 5–0 resorbable suture. Cranial bones were collected at eight weeks following surgery. Our animal experiments were approved by the Southern University of Science and Technology Yantian Hospital.

### 2.12. Histological Assessment

Mice were euthanized via injecting excessive pentobarbital sodium. The cranial bone defect specimens were fixed, decalcified, and dehydrated. Thereafter, the specimens were embedded in paraffin and sectioned into 5 *μ*m, followed by methylene blue and basic fuchsin staining. Sections were immunohistochemically or immunofluorescently stained, and antibodies included CD34 (1 : 100; ab81289; Abcam), LIF (1 : 100; ab113262), LIFR (1 : 100; ab232877), gp130 (1 : 100; ab259927), PI3K (1 : 100; ab32089), p-PI3K (1 : 100; ab182651), AKT (1 : 100; ab8805), p-AKT (1 : 100; ab38449), Nrf2 (1 : 200; ab62352), and GPx-3 (1 : 100; ab256470).

### 2.13. Statistical Analyses

Data were expressed as mean ± standard deviation. All analyses were conducted with SPSS 23.0 software. All experiments were repeated at least three times. Statistical difference between groups was determined with one-way analysis of variance. *P* values were labeled as follows: Ns: no significance, ^∗^*P* < 0.05, ^∗∗^*P* < 0.01, ^∗∗∗^*P* < 0.001, and ^∗∗∗∗^*P* < 0.0001.

## 3. Results

### 3.1. BMSCs Display Increased Apoptosis and Oxidative Stress and Reduced Mitochondrial Membrane Potential in Hypoxic Condition

To identify murine BMSCs, we examined cell surface antigens via flow sorting. In Figure 1(a), CD29-, CD44-, CD90-, CD105-, CD146-, and CD45-positive cells accounted for 95.27%, 99.01%, 99.84%, 99.88%, 40.49%, and 2.46%, respectively, suggesting that the isolated cells were BMSCs with high purity. Thereafter, BMSCs were exposed to 6 h-, 12 h-, and 24 h-hypoxic conditions for establishing hypoxic models. Both flow cytometry and TUNEL staining demonstrated that hypoxic BMSCs exhibited elevated apoptosis (Figures 1(b)–1(e)). Mitochondrial membrane potential was examined through by a JC-1 fluorescent dye, showing red fluorescence under aggregation condition in normal mitochondria as well as green fluorescence in decreased mitochondrial membrane potential. We noted that green fluorescence was increased as well as red fluorescence reduced in the hypoxic condition (Figures 1(f) and 1(g)). This conversion from red to green fluorescence indicated the reduction in mitochondrial membrane potential of BMSCs. Inactivation of Keap1/Nrf2 protects BMSCs from oxidative stress [25]. In the hypoxic environment, BMSCs displayed elevated Keap1 as well as reduced Nrf2 activity (Figures 1(h)–1(j)), indicating hypoxia-induced oxidative stress in BMSCs.

### 3.2. Increased LIF/LIFR/gp130 Activity and Reduced PI3K/Akt Activity in Hypoxic BMSCs

In the hypoxic condition, we examined the activity of LIF, LIFR, and gp130 in BMSCs. Under 6 h and 24 h hypoxic treatment, LIF, LIFR, and gp130 exhibited upregulation in BMSCs (Figures 2(a)–2(h)). Additionally, the reduction in PI3K, p-PI3K, AKT, and p-AKT activity was investigated in hypoxic BMSCs (Figures 2(i)–2(m)), indicating that hypoxia inactivated PI3K/Akt signaling in BMSCs. As expected, HIF-1*α* was upregulated in BMSCs with hypoxia exposure (Figure 2(n)). 6 h hypoxic exposure was utilized for subsequent experiments.

### 3.3. Upregulated LIF Alleviates Apoptosis and Oxidative Stress and Heightens Mitochondrial Activity and PI3K/Akt Signaling in Hypoxic BMSCs

LIF deficiency aggravated BMSC apoptosis with hypoxic condition; oppositely, LIF upregulations alleviated hypoxia-induced apoptosis in BMSCs (Figures 3(a)–3(d)). Moreover, further reduction in mitochondrial membrane potential of hypoxic BMSCs was found when LIF was knocked out (Figures 3(e) and 3(f)). Conversely, overexpressed LIF ameliorated mitochondrial activity of hypoxic BMSCs. Additionally, hypoxic BMSCs presented the increase in Keap1 as well as the reduction in Nrf2, SOD1, catalase, and GPx-3, which was exacerbated by LIF loss (Figures 3(g)–3(m)). LIF overexpression decreased Keap1 as well as heightened Nrf2, SOD1, catalase, and GPx-3 activity in hypoxic BMSCs, demonstrating that LIF enabled alleviating hypoxia-induced oxidative stress. Moreover, LIF and LIFR expression was further lessened in hypoxic BMSCs with LIF knockdown (Figures 3(n)–3(q)). Inversely, their expression was upregulated in hypoxic BMSCs when LIF was overexpressed. We also found that LIF loss further decreased the activity of PI3K, p-PI3K, AKT, and p-AKT but elevated HIF-1*α* expression in hypoxic BMSCs, with the opposite findings when LIF was overexpressed (Figures 3(r)–3(w)), demonstrating that LIF heightened PI3K/Akt signaling activation in hypoxic BMSCs.

### 3.4. Upregulated LIF Promotes Self-Renewal and Differentiation of Hypoxic BMSCs

Exogenous interference with LIF expression further impaired the proliferative capacity of BMSCs under hypoxia, while overexpressed LIF ameliorated the inhibitory effect of hypoxia on BMSC proliferation (Figures 4(a)–4(d)). In the hypoxic condition, cell surface antigens CD105, CD90, and CD29 presented decreased levels in BMSCs (Figures 4(e)–4(j)). The reduction in CD105, CD90, and CD29 levels was further aggravated by LIF knockdown. Nevertheless, upregulated LIF elevated their activity in hypoxic BMSCs. Hence, LIF motivated self-renewal and differentiation of hypoxic BMSCs.

### 3.5. LIF Upregulation Heightens the Osteogenic Differentiation of Hypoxic BMSCs

The activity of ALP, OCN, and BSP presented reduction in hypoxic BMSCs, while exogenous interference with the expression of LIF further reduced their activity (Figures 5(a)–5(f)). Overexpressed LIF alleviated the inhibitory effect of hypoxia on ALP, OCN, and BSP activity in BMSCs. Thus, LIF enabled heightening the osteogenic differentiation of BMSCs under hypoxic environment.

### 3.6. LIF Upregulation Alleviates Oxidative Stress in Hypoxic BMSCs through Activating PI3K/Akt Signaling

In the hypoxic condition, PI3K/Akt signaling agonist 740Y-P further elevated the levels of SOD1, catalase, and GPx-3 in BMSCs, with the opposite findings for PI3K/Akt signaling inhibitor LY294002 (Figures 6(a)–6(d)). Additionally, 740Y-P heightened the promoting effect of upregulated LIF on SOD1, catalase, and GPx-3 levels in hypoxic BMSCs; inversely, LY294002 impaired the promoting effect of upregulated LIF on their expression, demonstrating that LIF enabled alleviating oxidative stress in hypoxic BMSCs via heightening PI3K/Akt signaling activity. Our findings also demonstrated that PI3K, p-PI3K, AKT, and p-AKT expressions were activated by PI3K/Akt signaling agonist 740Y-P as well as lessened by inhibitor LY294002 in hypoxic BMSCs in the presence of LIF overexpression (Figures 6(e)–6(i)). Additionally, 740Y-P lessened HIF-1*α* activity in hypoxic BMSCs, with the opposite findings for LY294002 (Figure 6(j)). 740Y-P heightened the inhibitory effect of LIF on HIF-1*α* in hypoxic BMSCs, with the opposite findings for LY294002. Immunofluorescent staining demonstrated that LIF and LIFR expression was elevated by 740Y-P as well as decreased by LY294002 in hypoxic BMSCs (Figures 6(k)–6(n)).

### 3.7. LIF Upregulation Weakens Apoptosis and Ameliorates Mitochondrial Activity in Hypoxic BMSCs by Activating PI3K/Akt Signaling

In hypoxic environment, PI3K/Akt pathway agonist 740Y-P enhanced the inhibitory effect of LIF overexpression on BMSC apoptosis, while PI3K/Akt pathway-specific inhibitor LY294002 weakened the inhibitory effect of LIF overexpression on BMSC apoptosis (Figures 7(a)–7(d)). Furthermore, 740Y-P synergistically increased the mitochondrial membrane potential with LIF overexpression, while LY294002 attenuated the promoting effect of LIF overexpression on mitochondrial activity (Figures 7(e) and 7(f)). 740Y-P synergized with LIF overexpression to enhance Keap1 expression and decrease Nrf2 expression, with the opposite findings for LY294002 (Figures 7(g)–7(i)). Hence, LIF alleviated apoptosis and improved mitochondrial activity in hypoxic BMSCs via activating PI3K/Akt signaling.

### 3.8. LIF Improves Proliferation, Self-Renewal, and Differentiation of Hypoxic BMSCs by Activating PI3K/Akt Signaling

PI3K/Akt signaling agonist 740Y-P and LIF overexpression synergistically enhance BMSC proliferation under hypoxic conditions, with the opposite findings for inhibitor LY294002 (Figures 8(a)–8(d)). Moreover, the combination of 740Y-P and LIF upregulation heightened CD105, CD90, and CD29 levels in hypoxic BMSCs (Figures 9(a)–9(d)). Nevertheless, LY294002 impaired the promoting effect of LIF on their levels. It was also found that 740Y-P and LIF upregulation synergistically heightened ALP, BSP, and OCN activity in hypoxic BMSCs, with the opposite findings for LY294002 (Figures 9(e)–9(h)). Hence, LIF was capable of improving the proliferative capacity of hypoxic BMSCs by activating PI3K/Akt signaling.

### 3.9. Implantation of LIF-Overexpressed BMSC-Loaded BCP Scaffolds Increases Osteogenesis and Alleviates Oxidative Stress and Apoptosis through PI3K/Akt Signaling

We constructed a murine calvarial bone defect model that was implanted by LIF-overexpressed, PI3K/Akt signaling agonist 740Y-P or inhibitor LY294002 BMSC-loaded BCP scaffolds. After eight weeks, LIF-overexpressed BMSC-loaded BCP scaffolds remarkably increased the bone volume and bone density, which was synergistically enhanced by 740Y-P (Figure 10(a)). Nevertheless, LY294002 BMSC-loaded BCP scaffolds decreased the bone volume and bone density. Implantation of LIF-overexpressed or 740Y-P BMSC-loaded BCP scaffolds presented lower apoptosis, with the opposite findings for LY294002 BMSC-loaded BCP scaffolds (Figures 10(b) and 10(c)). Additionally, CD34 was upregulated when LIF-overexpressed or 740Y-P BMSC-loaded BCP scaffolds were implanted (Figures 10(d) and 10(e)). Oppositely, its expression was downregulated by implantation of LY294002 BMSC-loaded BCP scaffolds. It was also found that LIF, LIFR, gp130, PI3K, p-PI3K, AKT, p-AKT, Nrf2, and GPx-3 were upregulated following implanting LIF-overexpressed BMSC-loaded BCP scaffolds, which were synergistically enhanced by 740Y-P as well as weakened by LY294002 (Figures 11(a)–11(j)). Hence, implantation of LIF-overexpressed BMSC-loaded BCP scaffolds may elevate bone volume and bone density and alleviate apoptosis and oxidative stress via enhancing PI3K/Akt signaling activity.

## 4. Discussion

BMSC transplantation remains an available therapeutic regimen for bone defect restoration [26]. Nevertheless, during the transplantation process, the function and viability of BMSCs can be damaged because of extended duration of the in vitro culture, ageing, as well as patients' disease condition, etc. [27]. Severe hypoxia usually suppresses proliferation and osteogenic differentiation of BMSCs and impedes bone defect reconstruction [28]. In the treatment of large bone defects, ischemia and hypoxia in the bone defect area remain a thorny issue [29]. Here, hypoxic BMSCs presented increased apoptosis and oxidative stress and reduced mitochondrial activity. Enhanced mitochondrial activity triggers proliferative and migratory capacities along with osteogenic differentiation of BMSCs and thus facilitates bone defect repair [27]. In the hypoxic environment, BMSCs exhibited increased HIF-1*α* activity. Severe hypoxia induces HIF-1*α* accumulation and transfers into the nucleus, thereby reducing cellular proliferation and osteogenic differentiation of BMSCs [30]. Additionally, BMSC-exosomes carrying mutant HIF-1*α* can improve angiogenesis as well as osteogenesis in critical-size calvarial defects [31].

Our study demonstrated that LIF, LIFR, and gp130 were upregulated in hypoxic BMSCs. Upregulated LIF alleviated apoptosis and oxidative stress and heightened mitochondrial activity and PI3K/Akt signaling in hypoxic BMSCs. Controlling oxidative stress by activating antioxidant signaling is essential for bone homeostasis [32]. Keap1 can bind to nuclear factor Nrf2, a redox-sensitive transcription factor, thereby suppressing Nrf2 activation [33]. Nrf2 enhances the expression of multiple antioxidant and detoxification genes (SOD1, catalase, GPx-3) via antioxidant response elements [33]. Its loss triggers oxidative stress as well as facilitates RANKL-induced osteoclast differentiation [34]. Additionally, activated Nrf2 enhances the osteogenic ability of human dental pulp stromal cells via alleviating oxidative stress [35]. Our study showed the increase in Keap1 as well as the reduction in Nrf2, SOD1, catalase, and GPx-3 in hypoxic BMSCs, demonstrating that hypoxia induced oxidative stress in BMSCs. Upregulated LIF alleviated hypoxia-induced oxidative stress in BMSCs. Activated PI3K/Akt signaling also decreased Keap1 as well as elevated Nrf2, SOD1, catalase, and GPx-3 in hypoxic BMSCs, demonstrating that PI3K/Akt signaling activation enabled alleviating hypoxia-induced oxidative stress in BMSCs. Evidence suggests that PI3K/Akt-triggered Nrf2 signaling is capable of suppressing oxidative stress along with apoptosis in hepatic damage [36]. Suppressing PI3K/Akt signaling reversed the antioxidative stress of LIF in hypoxic BMSCs. Activated PI3K/Akt signaling heightens bone regeneration in critical-size defects [37]. Herein, LIF overexpression promoted self-renewal and osteogenic differentiation of BMSCs with hypoxic condition. Further, LIF enhanced self-renewal and differentiation as well as attenuated oxidative stress of BMSCs through upregulating PI3K/AKT signaling. In calvarial bone defect models, implantation of LIF-overexpressed BMSC-loaded BCP scaffolds enabled facilitating osteogenesis as well as alleviating oxidative stress and apoptosis through PI3K/Akt signaling.

Nonetheless, a few limitations should be pointed out. First, this study adopted BCP scaffolds, and other types of scaffolds for BSMCs will be considered in our future research, thereby improving the BMSC-mediated bone defect repair potential of LIF. Second, future research might extend the investigating duration to verify the beneficial effect of LIF on self-renewal and differentiation of BMSCs.

## 5. Conclusion

In conclusion, our work suggested the crucial role of LIF in promoting bone regeneration. Upregulated LIF might be a feasible approach for enhancing self-renewal and differentiation and attenuating oxidative stress of BMSCs in vitro via activating PI3K/AKT signaling, as well as bone defect repair in vivo. Thus, upregulated LIF in BMSCs offers great therapeutic promise for improving BMSC function and bone defect reconstruction.

## Figures and Tables

**Figure 1:** BMSCs exhibit increased apoptosis and oxidative stress along with reduced mitochondrial membrane potential in hypoxic condition. (a) Isolation and identification of BMSCs by detecting cell surface antigens via flow sorting. (b, c) Flow cytometry and (d, e) TUNEL staining for examining apoptosis of BMSCs under exposure to hypoxia for 6, 12, and 24 h. Bar, 20 *μ*m. (f, g) JC-1 staining for detecting mitochondrial membrane potential of hypoxic BMSCs. Bar, 20 *μ*m. (h–j) Immunoblotting of the activity of Keap1 and Nrf2 in hypoxia-exposed BMSCs.

**Figure 2:** Increased LIF/LIFR/gp130 activity and reduced PI3K/Akt activity in hypoxic BMSCs. (a–d) Immunoblotting of LIF, LIFR, and gp130 activity in BMSCs when exposed to hypoxia for 6, 12, and 24 h. (e–h) Immunofluorescent staining of LIF and LIFR activity in BMSCs under hypoxic condition. Bar, 20 *μ*m. (i–n) Immunoblotting of PI3K, p-PI3K, AKT, p-AKT, and HIF-1*α* expression in hypoxic BMSCs.

**Figure 3:** Upregulated LIF alleviates apoptosis and oxidative stress and heightens mitochondrial activity and PI3K/Akt signaling in hypoxic BMSCs. (a, b) Flow cytometry and (c, d) TUNEL staining for BMSC apoptosis with hypoxic exposure, along with knockout or overexpressed LIF. Bar, 20 *μ*m. (e, f) JC-1 staining for examining mitochondrial membrane potential of hypoxic BMSCs with knockout or overexpressed LIF. Bar, 20 *μ*m. (g–m) Immunoblotting of the activity of Keap1, Nrf2, SOD1, catalase, and GPx-3 in hypoxic BMSCs with knockout or overexpressed LIF. (n–q) Immunofluorescent staining of LIF and LIFR activity in BMSCs with hypoxic exposure, along with knockout or overexpressed LIF. Bar, 20 *μ*m. (r–w) Immunoblotting of the activity of PI3K, p-PI3K, AKT, p-AKT, and HIF-1*α* in hypoxic BMSCs with knockout or overexpressed LIF.

**Figure 4:** Upregulated LIF promotes self-renewal and differentiation of hypoxic BMSCs. (a, b) Colony formation and (c, d) EdU staining for examining BMSC proliferation with exogenous interference or overexpression of LIF under hypoxic condition. Bar, 20 *μ*m. (e–j) Flow sorting for detecting cell surface antigens (CD105, CD90, and CD29) in hypoxic BMSCs with LIF loss or overexpression.

**Figure 5:** LIF upregulation heightens the osteogenic differentiation of hypoxic BMSCs. (a–f) Immunofluorescent staining for ALP, OCN, and BSP activity in hypoxic BMSCs with exogenous interference or overexpression of LIF. Bar, 20 *μ*m.

**Figure 6:** LIF upregulation alleviates oxidative stress in hypoxic BMSCs through activating PI3K/Akt signaling. (a–d) Immunoblotting for SOD1, catalase, and GPx-3 activity in hypoxic BMSCs with LIF overexpression as well as PI3K/Akt signaling agonist 740Y-P or inhibitor LY294002. (e–j) Immunoblotting for PI3K, p-PI3K, AKT, p-AKT, and HIF-1*α* activity in hypoxic BMSCs with LIF overexpression as well as PI3K/Akt signaling agonist 740Y-P or inhibitor LY294002. (k–n) Immunofluorescent staining for LIF and LIFR in hypoxic BMSCs with LIF overexpression as well as PI3K/Akt signaling agonist 740Y-P or inhibitor LY294002. Bar, 20 *μ*m.

**Figure 7:** LIF upregulation weakens apoptosis and ameliorates mitochondrial activity in hypoxic BMSCs by activating PI3K/Akt signaling. (a, b) Flow cytometry and (c, d) TUNEL staining for BMSC apoptosis in hypoxic environment with LIF overexpression as well as PI3K/Akt signaling agonist 740Y-P or inhibitor LY294002. Bar, 20 *μ*m. (e, f) JC-1 staining for detecting mitochondrial membrane potential of hypoxic BMSCs with LIF overexpression as well as PI3K/Akt signaling agonist 740Y-P or inhibitor LY294002. Bar, 20 *μ*m. (g–i) Immunoblotting for Keap1 and Nrf2 activity in hypoxic BMSCs with LIF overexpression as well as PI3K/Akt signaling agonist 740Y-P or inhibitor LY294002.

**Figure 8:** LIF improves proliferative capacity of hypoxic BMSCs by activating PI3K/Akt signaling. (a, b) Colony formation and (c, d) EdU staining for examining BMSC proliferation in hypoxic BMSCs with LIF overexpression as well as PI3K/Akt signaling agonist 740Y-P or inhibitor LY294002. Bar, 20 *μ*m.

**Figure 9:** LIF improves the self-renewal and differentiation of hypoxic BMSCs by activating PI3K/Akt signaling. (a–d) Flow sorting for detecting cell surface antigens (CD105, CD90, and CD29) in hypoxic BMSCs with LIF overexpression as well as PI3K/Akt signaling agonist 740Y-P or inhibitor LY294002. (e–h) Immunofluorescent staining for ALP, BSP, and OCN expressions in hypoxic BMSCs with LIF overexpression as well as PI3K/Akt signaling agonist 740Y-P or inhibitor LY294002. Bar, 20 *μ*m.

**Figure 10:** Implantation of LIF-overexpressed BMSC-loaded BCP scaffolds increases bone volume and bone density and alleviates apoptosis via PI3K/Akt signaling. (a) Methylene blue and basic fuchsin staining for examining the bone volume and bone density of the murine calvarial bone defect with LIF-overexpressed, PI3K/Akt signaling agonist 740Y-P or inhibitor LY294002 BMSC-loaded BCP scaffolds. Bar, 20 *μ*m. (b, c) TUNEL for apoptosis in the murine calvarial bone defect with implantation of LIF-overexpressed, PI3K/Akt signaling agonist 740Y-P or inhibitor LY294002 BMSC-loaded BCP scaffolds. Bar, 20 *μ*m. (d, e) Immunofluorescent staining for CD34 in the murine calvarial bone defect with implantation of LIF-overexpressed, PI3K/Akt signaling agonist 740Y-P or inhibitor LY294002 BMSC-loaded BCP scaffolds. Bar, 20 *μ*m.

**Figure 11:** Implantation of LIF-overexpressed BMSC-loaded BCP scaffolds alleviates oxidative stress through PI3K/Akt signaling. (a–j) Immunohistochemical staining for LIF, LIFR, gp130, PI3K, p-PI3K, AKT, p-AKT, Nrf2, and GPx-3 expressions in the murine calvarial bone defect with LIF-overexpressed, PI3K/Akt signaling agonist 740Y-P or inhibitor LY294002 BMSC-loaded BCP scaffolds. Bar, 20 *μ*m.

## Data Availability

The datasets analyzed during the current study are available from the corresponding authors on reasonable request.

## Abbreviations

BMSCs: Bone marrow-derived mesenchymal stem cells
LIF: Leukemia inhibitory factor
Keap1: Kelch-like ECH-associated protein 1
Nrf2: Nuclear factor-erythroid 2-related factor 2
HIF-1*α*: Hypoxia-inducible factor 1*α*
SOD1: Superoxide dismutase 1
GPx-3: Glutathione peroxidase 3
ALP: Alkaline phosphatase
BSP: Bone sialoprotein
OCN: Osteocalcin.

## References

[1] Hirata H., Zhang N., Ueno M. (2022). Ageing attenuates bone healing by mesenchymal stem cells in a microribbon hydrogel with a murine long bone critical-size defect model. *Immunity & Ageing*.

[2] Wu D., Chang X., Tian J. (2021). Bone mesenchymal stem cells stimulation by magnetic nanoparticles and a static magnetic field: release of exosomal miR-1260a improves osteogenesis and angiogenesis. *Journal of Nanobiotechnology*.

[3] Hsu M. N., Huang K. L., Yu F. J. (2020). Coactivation of endogenous Wnt10b and Foxc2 by CRISPR activation enhances BMSC osteogenesis and promotes calvarial bone regeneration. *Molecular Therapy*.

[4] Song Y., Wu H., Gao Y. (2020). Zinc silicate/nano-hydroxyapatite/collagen scaffolds promote angiogenesis and bone regeneration via the p38 MAPK pathway in activated monocytes. *ACS Applied Materials & Interfaces*.

[5] Wan Z., Zhang P., Liu Y., Lv L., Zhou Y. (2020). Four-dimensional bioprinting: current developments and applications in bone tissue engineering. *Acta Biomaterialia*.

[6] Zhang C., Xia D., Li J. (2022). BMSCs and osteoblast-engineered ECM synergetically promotes osteogenesis and angiogenesis in an ectopic bone formation model. *Frontiers in Bioengineering and Biotechnology*.

[7] Li D., Yang Z., Zhao X. (2021). A bone regeneration strategy via dual delivery of demineralized bone matrix powder and hypoxia-pretreated bone marrow stromal cells using an injectable self-healing hydrogel. *Journal of Materials Chemistry B*.

[8] Tao H., Han Z., Han Z. C., Li Z. (2016). Proangiogenic features of mesenchymal stem cells and their therapeutic applications. *Stem Cells International*.

[9] Zhang Y., Lv J., Guo H., Wei X., Li W., Xu Z. (2015). Hypoxia-induced proliferation in mesenchymal stem cells and angiotensin II-mediated PI3K/AKT pathway. *Cell Biochemistry and Function*.

[10] Li X., Yuan Z., Wei X. (2016). Application potential of bone marrow mesenchymal stem cell (BMSCs) based tissue-engineering for spinal cord defect repair in rat fetuses with spina bifida aperta. *Journal of Materials Science. Materials in Medicine*.

[11] García-Sánchez D., Fernández D., Rodríguez-Rey J. C., Pérez-Campo F. M. (2019). Enhancing survival, engraftment, and osteogenic potential of mesenchymal stem cells. *World Journal of Stem Cells*.

[12] Liang Y., Zhou R., Liu X. (2021). Investigation into the effects of leukemia inhibitory factor on the bone repair capacity of BMSCs-loaded BCP scaffolds in the mouse calvarial bone defect model. *Journal of Bioenergetics and Biomembranes*.

[13] Zhao B., Peng Q., Wang D. (2022). Leonurine protects bone mesenchymal stem cells from oxidative stress by activating mitophagy through PI3K/Akt/mTOR pathway. *Cell*.

[14] Niu X., Xu J., Liu J., Chen L., Qiao X., Zhong M. (2020). Landscape of N6-methyladenosine modification patterns in human ameloblastoma. *Frontiers in Oncology*.

[15] Yang B., Chen Q. (2021). Cross-talk between oxidative stress and m6A RNA methylation in cancer. *Oxidative Medicine and Cellular Longevity*.

[16] Cai G. P., Liu Y. L., Luo L. P. (2022). Alkbh1-mediated DNA N6-methyladenine modification regulates bone marrow mesenchymal stem cell fate during skeletal aging. *Cell Proliferation*.

[17] Loriot Y., Marabelle A., Guégan J. P. (2021). Plasma proteomics identifies leukemia inhibitory factor (LIF) as a novel predictive biomarker of immune-checkpoint blockade resistance. *Annals of Oncology*.

[18] Zhang C., Liu J., Wang J., Hu W., Feng Z. (2021). The emerging role of leukemia inhibitory factor in cancer and therapy. *Pharmacology & Therapeutics*.

[19] Wu B., Li Y., Li B. (2021). DNMTs play an important role in maintaining the pluripotency of leukemia inhibitory factor-dependent embryonic stem cells. *Stem Cell Reports*.

[20] Berry M. F., Pirolli T. J., Jayasankar V. (2004). Targeted overexpression of leukemia inhibitory factor to preserve myocardium in a rat model of postinfarction heart failure. *The Journal of Thoracic and Cardiovascular Surgery*.

[21] Hunter C. A., Jones S. A. (2015). IL-6 as a keystone cytokine in health and disease. *Nature Immunology*.

[22] Ye S., Zhang D., Cheng F. (2016). Wnt/*β*-catenin and LIF-Stat3 signaling pathways converge on Sp5 to promote mouse embryonic stem cell self-renewal. *Journal of Cell Science*.

[23] Liang Y., Zhou Y., Jiang T., Zhang Z., Wang S., Wang Y. (2011). Expression of LIF and LIFR in periodontal tissue during orthodontic tooth movement. *The Angle Orthodontist*.

[24] Dong S., Zhen F., Xu H., Li Q., Wang J. (2021). Leukemia inhibitory factor protects photoreceptor cone cells against oxidative damage through activating JAK/STAT3 signaling. *Annals of Translational Medicine*.

[25] Yang N., Sun H., Xue Y. (2021). Inhibition of MAGL activates the Keap1/Nrf2 pathway to attenuate glucocorticoid-induced osteonecrosis of the femoral head. *Clinical and Translational Medicine*.

[26] Liu A., Lin D., Zhao H. (2021). Optimized BMSC-derived osteoinductive exosomes immobilized in hierarchical scaffold via lyophilization for bone repair through Bmpr2/Acvr2b competitive receptor-activated Smad pathway. *Biomaterials*.

[27] Guo Y., Chi X., Wang Y. (2020). Mitochondria transfer enhances proliferation, migration, and osteogenic differentiation of bone marrow mesenchymal stem cell and promotes bone defect healing. *Stem Cell Research & Therapy*.

[28] Fan D., Liu H., Zhang Z. (2021). Resveratrol and angiogenin-2 combined with PEGDA/TCS hydrogel for the targeted therapy of hypoxic bone defects via activation of the autophagy pathway. *Frontiers in Pharmacology*.

[29] Peng Z., Wang C., Liu C. (2021). 3D printed polycaprolactone/beta-tricalcium phosphate/magnesium peroxide oxygen releasing scaffold enhances osteogenesis and implanted BMSCs survival in repairing the large bone defect. *Journal of Materials Chemistry B*.

[30] Sha Y., Lv Y., Xu Z., Yang L., Hao X., Afandi R. (2017). MGF E peptide pretreatment improves the proliferation and osteogenic differentiation of BMSCs via MEK-ERK1/2 and PI3K-Akt pathway under severe hypoxia. *Life Sciences*.

[31] Ying C., Wang R., Wang Z. (2020). BMSC-exosomes carry mutant HIF-1*α* for improving angiogenesis and osteogenesis in critical-sized calvarial defects. *Frontiers in Bioengineering and Biotechnology*.

[32] Park M. W., Cha H. W., Kim J. (2021). NOX4 promotes ferroptosis of astrocytes by oxidative stress-induced lipid peroxidation via the impairment of mitochondrial metabolism in Alzheimer's diseases. *Redox Biology*.

[33] Yu C., Xiao J. H. (2021). The Keap1-Nrf2 system: a mediator between oxidative stress and aging. *Oxidative Medicine and Cellular Longevity*.

[34] Hyeon S., Lee H., Yang Y., Jeong W. (2013). Nrf2 deficiency induces oxidative stress and promotes RANKL-induced osteoclast differentiation. *Free Radical Biology & Medicine*.

[35] Zhang J., Li R., Man K., Yang X. B. (2022). Enhancing osteogenic potential of hDPSCs by resveratrol through reducing oxidative stress via the Sirt1/Nrf2 pathway. *Pharmaceutical Biology*.

[36] Rajendran P., Ammar R. B., Al-Saeedi F. J. (2021). Kaempferol inhibits zearalenone-induced oxidative stress and apoptosis via the PI3K/Akt-mediated Nrf2 signaling pathway: in vitro and in vivo studies. *International Journal of Molecular Sciences*.

[37] Yang C., Liu X., Zhao K. (2019). miRNA-21 promotes osteogenesis via the PTEN/PI3K/Akt/HIF-1*α* pathway and enhances bone regeneration in critical size defects. *Stem Cell Research & Therapy*.

